The article "Analysis of Therapeutic Effect of Elderly Patients with Severe Heart Failure Based on LSTM Neural Model" was retracted in 2023. Reasons: unreliable results or conclusions; lack of ethics approval or compliance; concerns about the data; concerns about the peer review.

# Analysis of Therapeutic Effect of Elderly Patients with Severe Heart Failure Based on LSTM Neural Model

**DOI:** 10.1155/2022/7250791

**Published:** 2022-08-28

**Authors:** Shunhong Chen, Shoudu He

**Affiliations:** Department of Emergency, Affiliated Hospital of Gansu University of Chinese Medicine, Lanzhou 730000, Gansu, China

## Abstract

In recent years, cardiovascular-related diseases have become the “number one killer” threatening human life and health and have received much attention. The timely and accurate detection and diagnosis of arrhythmias and heart failure are relatively common heart diseases, which are of great social value and research significance in improving people's quality of life by providing early treatment or intervention for those who are at risk. Based on this, this paper proposes a deep learning network architecture based on the combination of long- and short-term memory networks and deep residual neural networks for the automatic detection of heart failure. A total of 60 elderly patients with severe heart failure treated in the emergency department of our hospital from August 2019 to August 2021 were selected as the sample subjects of this study. The treatment outcomes and prognostic quality of life of the two groups of patients were compared and analyzed. Based on the unbiased test method, the accuracy of the proposed method on the authoritative open continuous heart rate database PhysioNet was 99.67% (data length 500), 98.84% (data length 1000), and 96.63% (data length 2000). This indicates that the network model can well extract the high-dimensional features of continuous heart rate and improve the accuracy of the classification model. The LSTM neural model proposed in this paper may be able to provide richer information on heart health status for portable ECG detection systems, which have very important clinical value and social significance.

## 1. Introduction

Population aging has always been a major social issue in China, and the results of the seventh census show that the total population of the country will be about 1.44 billion by the end of 2020, of which 18.7% will be 60 years old and above and 13.5% will be 65 years old and above [1], and the number of people suffering from cardiovascular diseases is increasing as the process of aging and urbanization accelerates, especially in the low-age and low-income groups. The potential risk factors for cardiovascular diseases show rapid growth and individual aggregation. Based on previous surveys, the report estimates that the number of people suffering from cardiovascular diseases in China has reached 290 million [2]. It is expected that the number of cardiovascular diseases will continue to show a rapid increase in the next decade [3].

There is more than one risk factor for cardiovascular disease, and most of the cases are due to the long-term superposition of several adverse factors that interact with each other, so we cannot make a one-sided analysis. Especially in recent years, it has been found that atmospheric pollution is also one of the risk factors for the development of cardiovascular diseases, especially PM2.5 as the main pathogenic component of particulate matter (PM), which has a closer relationship with cardiovascular diseases [4]. Since 2004, the average annual growth rate of total hospitalization costs for cardiovascular diseases alone has been much higher than the growth rate of gross domestic product (GDP) in the same period [5]. In summary, the prevention and treatment of cardiovascular diseases have become an important part of public health construction in China and have attracted the attention of the state and society.

In addition, the elderly are prone to diseases specific to this population and various complications and organ failure. The course of heart failure is shown in Figure 1. In addition, heart failure in the elderly has the following characteristics: the more women there are, the more the HFPEF is (also known as diastolic heart failure), the more patients have weakness, comorbidity and cognitive impairment, poor treatment outcomes, and mortality and hospitalization rates remain constant for years [6]. It is difficult to translate “evidence-based medical information” directly into evidence for the treatment of heart failure in the elderly because elderly patients with heart failure, particularly mental retardation, frailty, and comorbidities, fall under the exclusion criteria of clinical trials and have little evidence-based medical evidence. As a result, the prevention and treatment of elderly patients with heart failure are more complex and specific.

Studies have shown that heart failure can be detected based on quantitative indicators of continuous heart rate [7]. It was found that the standard deviation of continuous heart rate (SDNN) could be used to predict the risk of death in patients with heart failure [8]. Since then, researchers have been trying to identify heart failure patients by analyzing continuous heart rates. In recent years, deep learning algorithms have been continuously applied in various fields such as image recognition, speech analysis, and natural language processing with remarkable results [9]. Among the many deep learning models, the deep residual network (RESNET) [10] is particularly outstanding and is rapidly becoming one of the most popular network frameworks for various computer vision tasks. In this paper, we identify heart failure based on the deep residual network architecture and short-term continuous heart rate signals to effectively improve the accuracy and real-time performance of heart failure detection, help heart failure patients self-manage, improve survival and quality of life, and lay the foundation for more accurate and convenient heart health monitoring in the future.

## 2. Related Work

After more than 100 years of development, ECG testing equipment is now gradually improved, not only in terms of its shrinking size but also in terms of its clear recording and anti interference ability. In recent years, with the emergence and development of intelligent computers, people have also started to think whether they can use the power of computers to assist physicians in the observation and analysis of ECGs. Computer-Aided Diagnosis (CAD) system not only effectively solves the problem of subjective consciousness uncertainty that may occur during the analysis and diagnosis of ECG signals by doctors but also enhances the efficiency of doctors, which is of great practical significance to clinical work.

Among the machine learning algorithms, support vector machine (SVM) is one of the most frequently used methods for arrhythmia classification [11]. It has been reported that the 1-v-l (one-versus-one) SVM algorithm was used to classify ECG data and a high recognition rate is obtained. The authors in [12, 13] used the SVM classifier for the classification of six arrhythmias based on the ECG signal features extracted by the wavelet transform method and achieved an accuracy of 99.68%. Reference [14] et al. used the particle swarm optimization (PSO) algorithm to optimize the generalization performance of the SVM classifier and applied the system to the automatic classification of ECG signals and proved that the SVM approach outperformed other traditional classification algorithms, such as k-nearest neighbor (KNN) and radial basis function (RBF) neural networks. Reference [15] et al. then adopted a maximum voting strategy to hierarchically use SVM classifiers, thus improving the classification effect of SVM. Besides, some researchers also proposed a novel kernel function that significantly improved the final classification accuracy. However, the study also compared the classification results of the SVM-based algorithm with those of a deep learning network architecture based on a combination of long-term and short-term memory networks and deep residual neural networks and found that although the SVM algorithm outperformed the MLP method in terms of training time, the deep learning network architecture based on a combination of long-term and short-term memory networks and deep residual neural networks performed better in terms of accuracy, sensitivity, and so on. The performance is much better.

With the successful application of deep learning in other fields, more and more scholars have tried to use deep learning algorithms to solve practical problems in the field of ECG signal analysis [16]. Deep learning is an “end-to-end” approach, which makes predictions directly from raw data and can cope with a wider range of classification tasks. It can also improve the effectiveness of the learning process in the context of big data. Reference [17] in 2017 used Convolutional Neural Network for arrhythmia diagnosis based on single-lead ECG signals, which trained -a 34-layer convolutional neural network to detect arrhythmias in ECG time series of arbitrary length. Reference [18] et al. performed the classification of ECG signals based on deep neural networks, and the whole classification network was built using the current popular TensorFlow and Google toolboxes for the network. Reference [19], on the other hand, performed ECG signal classification based on the Alex Net deep learning architecture and achieved an average correct rate of 92%.

In summary, the relevance of deep learning network architectures based on a combination of long-term and short-term memory networks and deep residual neural networks to heart failure has been generally recognized by researchers, and the detection of heart failure using statistical methods or traditional machine learning methods has achieved some results, but there is still room for further improvement. The organic combination of deep learning and expert experience will be an important direction in this field in the future, and deep learning will also be the next hot spot for conducting heart failure diagnosis research due to its ability to extract high-dimensional features.

## 3. Experimental Data

The experimental data for this study were obtained from PhysioNet, an internationally recognized open-source database, which is divided into a clinical database and a waveform database. The waveform database contains continuous records of physiological signals in various noncritical care settings. In this study, we used the bidmc congestive heart failure database (bidmc-chf), the MIT-BIH normal sinus rhythm (NSR), and the fantasy database (FD).

The bidmc heart failure database included continuous ECG data of 15 patients with severe heart failure (NYHA grade 3-4), including 11 men aged 22 to 71 and 4 women aged 54 to 63; MIT-BIH normal sinus rhythm database includes continuous ECG data of 18 healthy people, including 5 men aged 26 to 45 and 13 women aged 20 to 50. The Fantasia database includes the physiological characteristics data of 20 young people (21 to 34 years old) and 20 elderly healthy subjects (68 to 85 years old) who have been strictly screened after 2 hours of rest. In this study, we first divide the database into a training set and a test set according to the subject's file information. The purpose of this is to ensure that the data in the test set never appear in the training stage and prevent the impact of overfitting on the algorithm evaluation. Then, the continuous heart rate data in the data set are divided into equal-length data with 500, 1000, and 2000 continuous heartbeats.  Table 1 summarizes the number of samples obtained from the above three databases after data segmentation.  Table 2 shows the information of subjects in the test set (there are many subjects in the training set, which are not listed here).  Figure 2 shows the schematic diagram of two kinds of continuous heart rate signals when the division length is 500 heartbeats.

## 4. Deep Network Structure

### 4.1. DBN Model

The DBN model consists of several layers of Restricted Boltzmann Machine (RBM) stacked on top of each other. An RBM contains visible and hidden layers, each layer consists of several neurons, and its structure is shown in Figure 3. In the RBM structure, neurons are interconnected between the visible and hidden layers, but there are no connections between neurons within each layer. The visible layer of the RBM satisfies the Bernoulli distribution or Gaussian distribution, while the hidden layer is the invisible feature detected and satisfies the Bernoulli distribution. The visible and hidden layers are connected by a symmetric weight matrix with probabilities satisfying the Boltzmann distribution.

For 1 set of values of (*v*, *h*) at a given state, assuming that both visible and hidden layer neurons obey Bernoulli distribution, the energy function can be expressed as

(1) $$\begin{array}{c} E\left(v,h,\theta \right)=-\sum_{i=1}^{m}\sum_{j=1}^{n}w_{ij}v_{i}h_{j}-\sum_{i=1}^{m}a_{i}v_{i}-\sum_{j=1}^{n}b_{j}h_{j}, \end{array}$$

where *θ*=*w*_*ij*_ is the connection weight between *v*_*i*_ and *h*_*j*_; *a*_*i*_ and *b*_*j*_ are the parameters of the RBM model; *v*_*i*_ is the *i* th neuron of the visible layer, corresponding to the investment of the *i* th item attribute; *h*_*j*_ is the *j* th neuron of the hidden layer; *m* and *n* are the number of neurons in the visible and hidden layers, respectively; and *a*_*i*_ and *b*_*j*_ are the unit biases of the visible and hidden layers, respectively.

The visible and hidden layers are independent of each other, and the conditional probability of *h* on *v* is

(2) $$\begin{array}{c} P\left(h|v\right)=\prod_{j}P\left(h|v\right). \end{array}$$

When *v*_*i*_ and *h*_*j*_ are given, the conditional probability distribution can be calculated as

(3) $$\begin{array}{c} \left\{\begin{array}{c} P\left(h_{j}=1|v;\theta \right)=\sigma \left(\sum_{i=1}^{m}w_{ij}v_{i}+a_{i}\right),\\ P\left(v_{j}=1|h;\theta \right)=\sigma \left(\sum_{j=1}^{n}w_{ij}h_{j}+b_{j}\right). \end{array}\right. \end{array}$$

The excitation function *σ* is chosen as the Sigmoid function.

(4) $$\begin{array}{c} \sigma \left(x\right)=\frac{1}{\left(1+e^{-x}\right)}. \end{array}$$

Given 1 set of defined training sets {*V*^*c*^*|c*{1,2,3 … *c*}}, the training objective is to maximize the log-likelihood function of the established model, and by calculating the gradient of the likelihood function, the weight update formula of the RBM can be obtained.

(5) $$\begin{array}{c} \Delta w_{ij}=\varepsilon \left(E_{\text{data}}\left(v_{i}h_{j}\right)-E_{\text{model}}\left(v_{i}h_{j}\right)\right), \end{array}$$

where *ε* is the learning rate; *E*_data_ is the expected output of the input data of the observation layer; and *E*_model_ is the expected output on the probability distribution of the model.

The DBN model consisting of multiple RBMs stacked bottom-up is shown in Figure 4. This deep confidence network is divided into 2 layers, the bottom DBN pretraining model and the top back propagation (BP) fine-tuning model, respectively.

### 4.2. Model Training Method

The traditional neural network uses the BP algorithm to train the network, but with the increase of the number of hidden layers, the BP algorithm has the problems of gradient gradually sparse and easy to converge to the local minimum. DBN based on deep learning can better solve the problems of the BP algorithm by pretraining and fine-tuning the network parameters, which is divided into the following 2 steps.

#### 4.2.1. Pretraining

Each layer of the network is trained separately and unsupervised, and the output of the upper layer is used as the input of the lower layer to ensure that as much information as possible is retained when the feature vectors are mapped to different feature spaces.

### 4.3. Fine-Tuning

The BP network is set up in the last layer of the DBN to receive the output of the RBM as its input, and the network is trained in a supervised manner to achieve top-down fine-tuning of the parameters.

Each layer of the RBM network can only ensure that the weights within its layer map optimally to the feature vectors in that layer, so the BP network also propagates the deviation information from the top-down to each layer of the RBM, fine-tuning the whole DBN network. The whole training process can be regarded as the initialization of the weights of the deep BP network, thus overcoming the disadvantage of the BP network of randomly selecting the initial values and falling into the local optimum, and the training time and convergence speed are significantly improved.

The residual network, a convolutional neural network proposed by four scholars from Microsoft Research, won the ImageNet Large Scale Visual Recognition Challenge (ILSVRC) in 2015 for image classification [20]. The residual network is characterized by its ease of optimization and its ability to improve accuracy by adding considerable depth. Its internal residual block uses jump connections to alleviate the gradient disappearance problem associated with increasing depth in deep neural networks and has been used with good results in practical applications. As shown in Tables 1 and 2, it directly skips one or more layers, thus introducing the data output of the previous layers to the input part of the later data layers.

The emergence of deep residual network structure effectively solves the degradation problem in deep learning because the residual network learns the residual function *f*(*x*)=*H*(*x*) − *x* rather than *H*(*x*). Although the two forms of objective functions can approximate the required function in principle, the difficulty of learning is not the same. In fact, after a lot of practical verification, the deep residual network has higher accuracy than other networks, such as VGGNet and GoogleNet.

### 4.4. Heart Failure Diagnosis Based on Deep Residual Network

As described above, the continuous heart rate signal itself is a time series signal, which has both spatial information and temporal information. Therefore, based on the deep residual network, we introduce long short-term memory (LSTM) units to extract the features of time series more effectively. As shown in Figure 5, the prototype of long-term and short-term memory units is a recurrent neural network (RNN). It improves the processing of time information of long-term time series by adding an input gate, memory gate, and forgetting gate. LSTM network is very suitable for classification, processing, and prediction tasks based on time series data and has been successfully applied in the fields of tourism time prediction and music generation. As shown in Figure 6, in this study, we use the LSTM network to replace the convolution network between residual blocks. We choose adaptive moment estimation (Adam) as the optimizer, and its parameter is set to the learning rate of 0.001, *β*1  = 0.9, and *β*2  = 0.999.  Figure 7 is our deep learning model architecture based on LSTM.

## 5. Experimental Results and Analysis

### 5.1. Evaluating Indicator

In this study, we used accuracy, sensitivity, and specificity as validation indicators. The specific definitions are as follows:

(6) $$\begin{array}{c} Se=\frac{TP}{TP+FN}\text{specificity},\\ Sp=\frac{TN}{TN+FP}\text{accuracy},\\ Acc=\frac{TN+FP}{TP+FN+TN+FP}. \end{array}$$

It should be noted that in medical diagnosis, sensitivity refers to the ability of the algorithm to correctly detect patients with a certain disease, while specificity refers to the ability of the algorithm to correctly identify people without a disease.

### 5.2. Experimental Result

In practical clinical application, whether a model is mature and effective mainly depends on whether it can make accurate and reliable detection when facing patients. Therefore, in this study, we use the unbiased test to evaluate the effectiveness of the algorithm.  Table 3 shows the performance of this method on the unbiased test set.

Compared with the traditional heart failure recognition algorithm, the heart failure recognition algorithm based on deep learning can extract reliable features in high-dimensional space without manual operation and avoid possible human errors. Deep learning system finds the distributed feature representation of data by combining low-level features, so as to form a more abstract feature representation.

Figure 8 shows that after heart failure and cure, this method has two advantages. First, heart failure is detected based on the residual neural network. The decision system based on this method can automatically obtain useful information from all data, rather than manual data dimensionality reduction through feature extraction. This can preserve the useful information of the data to the greatest extent and avoid potential errors; Secondly, we modify the network architecture based on the LSTM network unit to make the model more suitable for the classification of time series signals. However, this study also has some limitations. Firstly, this study did not carry out multiclassification identification of heart failure with different severity and did not deeply discuss the effect of heart failure drugs on the continuous heart rate of subjects in the database. Secondly, this method needs big data to train the model to obtain the best performance, and the calculation consumption of the modified network model based on LSTM in the training stage is low.

## 6. Case Analysis

### 6.1. General Information

A total of 60 elderly patients with severe heart failure treated in the emergency department of our hospital from August 2019 to August 2021 were selected as the sample objects of this study. The selected patients were randomly divided into 30 patients in the control group who received only ordinary treatment and 30 patients in the observation group who received combined treatment. There were 19 male patients and 11 female patients in the control group, aged 49–71 years, with an average age of (61.3±7.1) years. There were 17 male patients and 13 female patients in the observation group, aged 48–80 years, with an average age of (62.1±6.9) years.

### 6.2. Observation Index

The treatment efficiency of the two groups was compared and analyzed. The higher the score, the higher the patient's score, and the better the quality of life.

## 7. Results

It can be seen from Table 4 that compared with the control group only receiving routine treatment, the curative effect of the observation group receiving combined treatment intervention is better, which is statistically significant (*P* < 0.05).

It can be seen from Table 5 that the prognosis and quality of life of patients in the observation group treated with combination therapy are significantly better than those in the control group treated only with routine therapy, and the difference between the two groups is statistically significant (*P* < 0.05).

## 8. Discussion

The main cause of severe heart failure is the myocardial strain caused by the patient's cardiomyopathy, myocardial infarction, and other hemodynamics with a large load, which changes the structural properties of the patient's myocardial function, and finally leads to the change of a cardiac function. Patients often show dyspnea and fatigue in the clinic, which not only reduces the quality of life of patients but also poses a threat to their life, health, and safety of patients. Therefore, timely and effective treatment for patients with severe heart failure is of positive significance to ensure the life safety of patients. During routine treatment, as *β* Metoprolol, a receptor blocker, can reduce blood pressure and control the patient's heart rate [21], which can effectively control the catecholamines secreted in the patient's body and slow down the myocardial damage, but it can not effectively improve the level of LVEF and fundamentally treat the heart problems of patients with heart failure. The addition of irbesartan hydrochlorothiazide on the basis of ordinary treatment can greatly improve the therapeutic effect. Irbesartan hydrochlorothiazide is an angiotensin II receptor inhibitor, which can effectively inhibit the activity of angiotensin, so as to reduce the incidence of hypokalemia and improve the actual treatment effect. Combined with the survey and research results, the treatment effective rate of the observation group was 96.67%, while that of the control group was 66.67%, and the quality of life score of the observation group was significantly higher than that of the control group (*P* < 0.05).

To sum up, in the treatment of elderly patients with severe heart failure, metoprolol combined with erbesar is more effective, can effectively improve the clinical symptoms and improve the quality of life of patients, and is worthy of popularization and application.

## 9. Conclusions

The proposed method is evaluated based on three open-source databases and four input data of different lengths. The results show that the accuracy of this method reaches 99.67%, 98.84%, and 96.63%, respectively, when the length is 500, 1000, and 2000. Heart failure detection using continuous heart rate is very important for medical and healthcare applications, especially for wearable devices such as smartwatches and bracelets. In the next step, we will deploy this model to healthcare applications as an auxiliary means for daily monitoring of patients with heart failure and try to add an attention mechanism to further improve the accuracy.

## Figures and Tables

**Figure 1:** Heart failure process.

**Figure 2:** Two types of data when the sample length is 500 heartbeats.

**Figure 3:** RBM model.

**Figure 4:** DBN.

**Figure 5:** Schematic diagram of the residual building block.

**Figure 6:** LSTM cell structure.

**Figure 7:** Deep network architecture.

**Figure 8:** Heart failure and post cure.

**Table 1:** Sample size of different databases.

Database		Split length	
	500	1000	2000
BIDMC-CHF	3214	1607	803
NSR	3579	1793	869
FD	500	250	125

**Table 2:** Information of subjects in the test set.

Subject information		Split length		
54,F,#11	50,F,#19830			
63,M,#13	38,F,#19140	686	339	164
61,M#14	34,M,#19093			

**Table 3:** Performance on unbiased test sets.

Signal length	Accuracy (%)	Sensitivity (%)	Specificity (%)
500	99.67	99.34	100
1000	98.84	97.53	100
2000	96.63	100	93.64

**Table 4:** Comparison of treatment effectiveness between the two groups.

Group	Number of cases	Remarkable effect	Effective	Invalid	Effective rate (%)
Control group	30	16	4	10	20 (66.67)
Observation group	30	26	4	1	29 (96.67)
*x* ^2^	-	-	-	-	9.017
*P*	-	-	-	-	0.003

**Table 5:** Comparison of quality of life scores between the two groups.

Group	Number of cases	Physiological function	Psychological function	Social function	Total score
Control group	30	48.62±8.32	60.41±11.71	61.64±9.32	58.75±6.32
Observation group	30	60.69±8.19	75.36±10.57	76.95±9.53	68.33±8.58
*T*	-	5.663	5.191	6.291	4.924
*P*	-	0.000	0.000	0.000	0.000

## Data Availability

The experimental data used to support the findings of this study are available from the corresponding author upon request.
